# Investigation of Factors Affecting COVID-19 and Sixth Wave Management Using a System Dynamics Approach

**DOI:** 10.1155/2022/4079685

**Published:** 2022-11-26

**Authors:** Nasser Safaie, Maryam Kaveie, Siroos Mardanian, Mina Mohammadi, Rasoul Abdol Mohamadi, Seyed Amir Nasri

**Affiliations:** Department of Industrial Engineering, K. N. Toosi University of Technology, Tehran, Iran

## Abstract

The COVID-19 pandemic has plunged the world into a health and economic crisis never seen before since the Spanish flu pandemic in 1918. The closure of schools and universities, the banning of rallies, and other social distancing in countries have been done to disrupt the transmission of the virus. Governments have planned to reduce restrictions on corona management by implementing vaccination programs. This research aims to better understand the Coronavirus disease's behavior, identify the prevalent factors, and adopt effective policies to control the pandemic. This study examines the different scenarios of releasing the constraints and returning to normal conditions before Corona to analyze the results of different scenarios to prevent the occurrence of subsequent peaks. The system dynamics approach is an effective means of studying COVID-19's behavioral characteristics. The factors that affect Coronavirus disease outbreak and control by expanding the basic SEIR model, interventions, and policies, such as vaccination, were investigated in this research. Based on the obtained results, the most critical factor in reducing the prevalence of the disease is reducing the behavioral risks of people and increasing the vaccination process. Observance of hygienic principles leads to disruption of the transmission chain, and vaccination increases the immunity of individuals against the acute type of infection. In addition, the closure of businesses and educational centers, along with government support for incomes, effectively controls and reduces the pandemic, which requires cooperation between the people and the government. In a situation where a new type of corona has spread, if the implementation of the policy of reducing restrictions and reopening schools and universities is done without planning, it will cause a lot of people to suffer.

## 1. Introduction

On December 31, 2019, COVID-19 was identified in Wuhan, China. With the Coronavirus disease outbreak and its high transmission rate, China quarantined the city of Wuhan and took strict measures to prevent the further spread of the virus to other parts of the country. Nevertheless, on March 11, 2020, COVID-19 was declared a global pandemic by the World Health Organization (WHO) due to its rapid spread to other parts of the world. According to reports, 118,000 positive cases were reported in 114 countries on the mentioned date, and about 4,000 people lost their lives. The WHO issued statements on the outbreak, calling all countries to take control measures to deal with the world's biggest-ever public health emergency. The first case of Coronavirus disease in Iran was officially announced on February 18, 2021. The government initially tried to control and fight against the unknown virus by closing schools and universities. Over time, new restrictions were imposed, but the apparent decrease in patients convinced the authorities to reduce the restrictions.

On the other hand, the reduction of health protocols, taking the disease for granted, and the adoption of wrong policies again increased the number of patients, so Iran passed the fourth peak of the disease and is now dealing with the fifth wave of the pandemic. The government has implemented various policies to prevent and reduce the incidence of COVID-19, but these policies have not been sufficient or have been poorly implemented. As of January 17, 2022, the number of patients in Iran and worldwide was about 6,221,000 and 329,000,000, respectively. Also, COVID-19 has taken the lives of some 132,000 people in Iran and 5,557,000 patients worldwide.  Table 1 shows information about patients, recoveries, and deaths from the beginning of the coronavirus disease outbreak until mid-January 2022 worldwide.

Virologists have conducted extensive studies on the virus genome to discover effective drugs for treating coronavirus disease patients. However, according to the Ministry of Health, no drug has been 100% effective in treating the disease. On the other hand, vaccination has always been one of the fundamental ways to deal with the pandemic. Therefore, with extensive research, several countries have successfully produced effective vaccines against the disease. According to the latest global statistics on coronavirus disease vaccination, until the first of 2022, 9 billion 326 thousand 391 doses of COVID-19 vaccine have been injected in different countries, among which in terms of the highest percentage of the vaccinated population, China stands at 86.1%, the USA at 62.9%, and India at 48%. The statistics of vaccine injections in Iran are about 60 million and 490 thousand first doses, 53 million and 586 thousand second doses, and around 14 million and 563 thousand third doses by January 23, 2022.

Although published statistics such as Figure 1 show that not all vaccines discovered are 100% safe against COVID-19, they noticeably reduce the incidence of the acute form leading to death. Although mutations in the primary virus may reduce the vaccine's effectiveness, vaccination is the best way to increase human immunity and reduce the costs associated with coronavirus disease.

The first mutation of the coronavirus disease, the alpha variant, known as the British Corona, was identified in September 2020 in southeast Britain. The new coronavirus disease entered and adhered to the respiratory cells, causing the virus to observe a higher transmission rate and faster spread. The first case of British Corona in Iran was recorded on January 4, 2021. The Alpha variant is so far spread across the UK and at least 70 countries. Another variant of the coronavirus disease mutation beta virus was first spread in October 2020 in South Africa. Beta has now spread throughout South Africa and more than 30 other countries. A new type of disease, the delta variant, spread in India in October 2021 and became more widespread with two mutations in the virus genome. An important feature of the Delta variant is its very high transmission rate, which is 60% higher than the alpha variant. Patients with the infection have been found in more than 80 countries. Researchers still do not know whether the delta strain causes more severe disease and is more deadly than other variants and how effective are the available vaccines?

Studies have shown that existing vaccines are still effective against mutated strains of the coronavirus disease, including the delta variant. The world is currently facing another type of coronavirus disease. The virus, called lambda, was first seen in Peru and has been reported in at least 40 countries. This is a substantially more contagious mutation than the Corona Delta. It is also highly resistant to antibodies and causes more infections than the alpha and delta variants. Lambda is three times more resistant to the vaccine and is more common in people with chronic diseases. No case of this variant has been observed in Iran yet. Another strain of the disease, called Mu, was first identified in January 2021 in Colombia, South America. This strain is now recognized in 39 countries, including the United States and European countries. The Mu variant has several characteristics that make it more resistant to vaccines, but more research is needed to understand its features better.

In November 2021, the World Health Organization (WHO) warned of a new strain of the coronavirus disease called Omicron. This species was first reported to the WHO in South Africa. Evidence suggests that Omicron has a number of mutations that affect how it behaves, such as the rate at which it spreads or the severity of the disease it causes. It is also predicted that this variable will reduce the effectiveness of public and social health measures or existing diagnoses, vaccines, and treatments. In less than a month after the official report, Omicron has spread to more than 100 countries, such as Canada, the United States, Spain, France, India, and so on.  Figure 2 shows the countries that have been infected with the virus. A study of Omicron infections shows that this type has a shorter incubation period. After contact with the infected person, it takes less than three days for the symptoms to appear in the person and the test result is positive. The first case of coronary heart disease in Iran was registered on December 19, 2021. Since then, 1162 people have been infected with this variant, and three people have lost their lives.

Figure 3 shows this variant spread more rapidly than others and is expected to become a common variant in the entire world in a short time. While COVID-19 is still prevalent around the world, some countries have decided to remove COVID restrictions, such as wearing masks, not holding rallies, and closing schools and universities, after implementing a vaccination plan and increasing the vaccinated population, reducing the number of cases and deaths. Therefore, with the advent of the new Omicron variant, infection rate and morbidity and mortality rates will rise. France and South Korea, for example, repealed hygiene, telecommuting, and anti-assembly laws after 75% and 84% vaccination, respectively. Still, with the outbreak of the new Omicron variant, the number of COVID-19 patients in these countries has increased. Governments sought to impose new restrictions, requiring employees to do their work at home if possible.  Figure 4 shows a diagram of daily infection cases in France, South Korea, and other countries. The European governments are worried about the fourth Corona peak in these areas. According to Figure 4, the incidence of the disease in some countries is increasing with a steep slope.

Concerns have risen internationally due to the high prevalence and consequent increase in deaths from COVID-19 disease.

Figure 5 represents the rate of decline of corona disease after the sixth wave; the decreasing trend of this graph can be a promise of the end of this disease in Iran. According to the figure, the sixth wave of this disease started in January 2022, and with a steep increase on February 8, 2022, we have witnessed the peak and highest death rate in this wave. The disease process is improving after the peak; so the number of deaths caused by Coronavirus disease is decreasing and fortunately, the statistics of this variable have tended to zero.

In addition to virologists, researchers in other fields have studied the COVID-19 pandemic from various perspectives. Some researchers have used mathematical modeling and simulations to understand the dynamics of the pandemic to provide valuable advice to physicians and politicians. One of the tools is to simulate the system dynamics approach, which focuses on the feedback behavior of variables in the closed-loop of the system and deals with how the behavior of internal feedback loops creates behavior in the system structure. The power of system dynamics lies in analyzing the impact of information feedback on decision-making in a complex system. Detailed modeling methods such as systems dynamics can be used to illustrate the dynamics of the outbreak and to simulate disease behavior with explicit assumptions. Public health practitioners believe that systemic approaches, such as systems dynamics, are valuable when developing effective policies.

In a study, researchers at the beginning of the COVID-19 pandemic used a dynamic system to model effective behaviors and policies for corona outbreak and control. The effect of factors such as quarantine, hospital availability, the proportion of hospital beds for corona patients, visits between sick and susceptible people on the number of infections, and deaths due to COVID-19 were investigated. They also reviewed the model results by presenting different scenarios. In other studies, various arrangements such as travel bans, social distancing, masks, telecommuting, and the closure of commercial centers were introduced to control the spread of the disease and prevent new cases of infection [1].

As mentioned above on the benefits of using SD in the behavior of epidemic diseases, in this study, we were able to better identify the factors affecting the prevalence and control of this disease with the effective use of the dynamic system. The purpose of this study was to investigate the outbreak of COVID-19 by removing the restrictions simultaneously with the emergence of a new Omicron variant in the world to examine the different scenarios for implementation of this decision and show the results to prevent acute diffusion conditions. In this study, the data from Iran has been used to examine the model. It was selected as the case study because it had access to the vaccine later due to sanctions against some countries and faced many difficulties in the preparation of the vaccine. In addition, due to the many national-religious ceremonies in this country, the impact of communities and health reduction principles in increasing the incidence of this disease can be well studied. Also, by examining the trend of previous peaks, it was observed that with the decrease in the number of patients and deaths due to coronary disease and psychological pressure affected by reduced social communication and staying at home, gatherings increased, and the country faced the next peak. Therefore, the results and scenarios were designed by examining the patients' information and deaths in Iran. In the proposed model, we look at the conditions of Omicron release in Iran by taking into account the booster dose.

By studying the previous researches and examining the Corona conditions of the Iranian society, a dynamic system model was presented in this research. The innovations of the proposed model are as follows:

- Considering vaccination in modeling
- Investigating the effect of vaccination on R0
- Adding parameters affecting the vaccination rate according to Iran's conditions, for instance: import of vaccines, access to vaccine
- With the increasing trend of people contracting the disease and the increase in new patients, booster dose injections have been considered in the proposed model
- Simultaneous consideration of the parameters that have directly or indirectly affected the rate of disease outbreak, such as supportive income, business closure, and economic pressure, can be mentioned.
- Predicting the occurrence of the sixth wave due to the reduction of observance of health principles and providing management solutions.

This paper suggested a comprehensive and integrated model that can simultaneously consider the three basic factors of service capacity facilities and the social and economic dimensions in the behavior of the people in the society in predicting the pandemic disease. These factors are among the important and effective parameters in changing the spread of a pandemic that in literature is ignored. Therefore one of our motivations in this study is to cover this gap.

Existing studies that utilize various approaches in analyzing the behavior of epidemic diseases have been examined in the literature review section. The research method and modeling algorithm are described in Section 3. In Section 4, the developed model and the stock-flow diagram of the proposed model are described in detail. In Section 5 of the working method, the model and research data formulation is presented. The validity of the suggested model will also be investigated by comparing the historical data method with the extreme condition test in Section 6.  Section 7 presents the sensitivity analyses, while Section 8 presents the different scenarios for the developed model.  Section 9 describes the scenario analysis. is the last part. It shows the proposed model results and makes suggestions for how to improve the model and make it work better in the real world. Then the last section describes the results of the proposed model and makes suggestions for how to improve the model and make it work better in the real world.

## 2. Literature Review

COVID-19 disease is a contagious disease that has caused much damage in various dimensions. More than four million people have died since the outbreak through mid-September 2021.

By examining the conditions of the Iranian society due to the sanctions and the late conclusion of the experiments related to the production of the vaccine in the fourth wave and the emergence of the delta strain, the number of infected increased sharply. At this time, the efforts of the Iranian government and the Ministry of Health, due to the lack of sufficient access to the vaccine and also based on the experiences gained from previous waves, to reduce the intensity of the upcoming waves, focused more on observing health principles and increasing social distance. In their paper, the researchers also focused on identifying factors affecting the outbreak, and in a limited number of studies, vaccination was considered. Also, in the investigated researches, factors affecting the prevention of outbreaks, such as supportive income, social distance, hospital capacity, etc., have not been considered at the same time. Also, many researches ignore the impact of vaccination on the outbreak rate. Therefore, by studying the circumstance of the number of patients after vaccination in other countries, in this research, the effect of vaccination and the factors affecting the vaccination rate in Iran were investigated, and the effect of the mentioned factors such as supportive income and social distance, etc., was considered simultaneously in this study.

The prevalence of the COVID-19 crisis has focused the attention of experts in various fields on finding a way to contain the crisis and study and control people's behavioral responses to the disease. Understanding the system's behavior is vital to providing appropriate planning to deal with the spread of epidemics [2]. In this regard, understanding the dynamics of the prevalent disease's behavior is critical for preparing health systems, equipment, and medical personnel. In recent years, the use of mathematical and statistical models, simulations, artificial intelligence, and data mining has helped us understand how epidemic diseases spread. This has helped us come up with effective ways to prevent and control the spread of such diseases. In the literature, extensive studies with a mathematical modeling approach have been conducted to investigate the effects of COVID-19 from various viewpoints. The mathematical model–based analysis is a powerful tool for understanding how the disease is transmitted and applying cost-benefit analysis in various functional scenarios. In this regard, many articles have reviewed various strategies to reduce the disease and its parameters for scenario-based analysis and active control methods to fight against COVID-19 disease. These articles give an overview of important epidemiological factors, such as how easy it is to spread, what happens when people move away from each other, how bad the disease is, how many people die from it, and so on.

One of the basic challenges in the development of human societies is to predict the real world in the future [3]. Because system dynamics (SD) analysis is a very efficient and well-known method for studying system behavior in disease outbreaks, researchers have used it to study the behavior of pandemic diseases. A study stated that the system dynamics modeling method is suitable for studying health issues and predicting the underlying systemic behavior. The possibility of using feedback, preparing scenarios, and analyzing the system's sensitivity to any factors involved are reasons for the tool's effectiveness [4]. A study presented one of the first system dynamics models as a new way of understanding how complex health care systems work. Since then, applying system dynamics or systems thinking to the study of public health services has been successful [5]. In studies performed on patients who initially develop the disease, after a while, the symptoms appear, and then they are treated. This method of examining patients is known as the susceptible, infected recovery (SIR) model [6–8]. In this model, the disease is transmitted during an incubation period. However, in some diseases, especially those that have spread in recent years, such as SARS in 2002 and COVID-19 in 2019, the disease appears after an incubation period, and in that period, the patient is rarely a carrier. For such diseases, it is necessary to review the SIR models again and develop SEIR [1] models accordingly. In the next section, we will look at the studies that were done to figure out how and how much COVID-19 is spread using the methods we have already talked about. This will help us group the models that are already out there.

## 3. Mathematical Models for COVID-19

In a study, they formulated a mathematical model for avian influenza and investigated the essential dynamics of the model through an equilibrium analysis [9]. By studying COVID-19 patients in India, the effects of social distancing and quarantine were analyzed, and coronavirus disease control strategies were examined using the SEQIR (S-Susceptible, E-Exposed, Q-Quarantine, I-Infected, R-Recovered) model [10]. In a study on epidemic evolution in Wuhan, China, a mathematical model evaluated the epidemiological features of the virus. The result showed that while Chinese intervention has effectively controlled the transmission of the disease, sustained global efforts are needed to contain the pandemic [11]. A study highlighted the role of mathematical modeling in COVID-19. It examined the challenges related to data availability, uncertainty, and the application of modeling-based approaches to help make decisions to control the disease [12]. An article presented a mathematical model for evaluating COVID-19 behaviors under different scenarios. It is discussed that scenarios can be an effective tool for convincing the society of the need for a comprehensive effort to reduce the prevalence of the disease. Also, by investigating different scenarios, it was observed that the application of quarantine and social distancing strategies has a remarkable effect on reducing the disease [13]. In another study, an SEIR-based model was proposed to predict the prevalence of the disease by considering existing policies such as transportation restrictions, reduced service levels, and social distancing [14]. An advanced model based on the SUQC [1] approach was developed using daily data to estimate the prevalence rate in Wuhan and four other cities in China [15]. A study using data from Brazil modeled the early evolution of the COVID-19 pandemic and predicted that the government's social distancing policy could control the prevalence of COVID-19 [16]. A study is presented using mathematical modeling and nonstandard to analyze and assess the impacts of environmental factors on Avian Influenza Virus type A infection. This model is formulated in terms of the nonlinear ordinary differential system [17]. Examining a new advanced SIV [2] model concerning known aspects of coronavirus disease behavior for the COVID-19 pandemic, a study established that with the help of simulation and susceptibility analysis, the sensitive parameters of the model have a more significant impact on disease prevalence and can be identified and controlled [18]. These parameters significantly reduced the number of patients and thus inhibited the disease. Using a mathematical model, another paper examined the relationship between control measures such as mask use and social distancing during the COVID-19 pandemic and economic reopening time [19]. Also, a model is formulated in the form of a system of differential equations, where the population is included in seven compartments: susceptible population, exposed, asymptomatic infection population, symptomatic infection population, recovered population, susceptible populations previously infected, and a quarantined population. According to the results, the outbreak will lessen if a strict social distancing policy is enforced like a quarantine [20].

### 3.1. COVID-19 Dynamics Models

System dynamics can be adopted as an approach to the behavior evaluation of the COVID-19 pandemic [21]. With the emergence of COVID-19 at the beginning of 2019, many studies attempted to model the factors affecting the prevalence and control of the disease and its effect on various aspects of life using the systems dynamics approach [22]. A study using systems dynamics modeling investigated the conditions of coronavirus disease inhibition in Iran. In Indonesia, to predict the peak of COVID-19, it was shown that considering various intelligent scenarios will strengthen the system's forecasting result. The study showed that observing social distancing, implementing health protocols, adequacy of health facilities and medical equipment, spraying, disinfection, quarantine, or telecommuting can reduce the development of the disease [23]. In China, by estimating the system parameters from the Particle Swarm Algorithm (PSO) according to the data of Hubei Province, they presented the SEIR model for modeling and predicting the condition of COVID-19 disease. In this study, quarantine has been described as the most effective way to control the disease [24]. An article presenting a dynamic model for the prevalence of COVID-19 disease predicted the impact of policies such as social distancing in different scenarios [25]. In Spain, they used SD data to develop an SD simulation model to examine proposed policies in STELL software [26]. In Iran, COVID-19 was studied using the SEIR-based system dynamics method and the available data in the country. As of March 20, 2020, the cumulative infected patients were estimated at 916,000, and the death toll was 15,485 [27]. In their study, they investigated the effects of therapeutic interventions and preventive measures on the coronavirus disease pandemic using a system dynamics approach based on the SEIR model. The proposed model analyzed the effects of people's behavior, contact with them, and general quarantine on the spread of the disease. Using data collected by the Iranian Ministry of Health, they examined the effect of hospital limitations and public health capacity on the rate of transmission and death. The study results showed that interventionist policies play an essential role in reducing the infection rate and the number of deaths, and thus, controlling the pandemic [28]. A dynamic system model is used to examine policy innovation, the emergence of innovative health technology, and their implications for a health system. The mixing of public health decisions and economic interests makes it hard to put innovation policy into action. This leads to the development of new health technologies that require the health system to be improved [29]. Organizations in charge of health need to implement blockchain technology because the blockchain platform guarantees that no part of the information is changed, so the checks and results are true [30]. Nowadays, disease control like COVID-19 requires different management methods. Machine learning, artificial intelligence, and information science have a great contribution in the fight against this disease [32]. Therefore, blockchain technology can help humanity in the fight against diseases such as COVID-19 by implementing a blockchain-based platform that connects local hospitals and health organizations in infected areas to those that are being infected, recording medical data of patients who have certain symptoms and examining these data to predict the spread of the virus, etc. These are the advantages blockchain technology brings [31], and machine learning techniques have been proposed to predict the death rate of corona patients in India, and based on the results, it has been proven that the proposed model performs better compared to other models such as support vector machine(SVM), decision tree, etc. [33]. Jamil et al. (2021) presented a comprehensive analysis of the socioeconomic effects of COVID-19 on public health through data mining strategies including correlation coefficient matrix, ARIMA, data mining techniques, decision trees, and statistical performance evaluation for the development of predictive models in Iran. The socioeconomic effects of this pandemic were investigated through quantitative analysis of stock market index, money inflation, gasoline price, interest rate, consumer price index, and crude oil price. Also, with the correlation matrix, they discovered the nature and intensity of interdependence of these features and finally developed a regression estimation model to predict the values of features related to each other [34].

A systematic review on COVID-19 demonstrates automated artificial intelligence applications based on data mining and machine learning (ML) algorithms to diagnose COVID-19 [35]. By examining the increasing exponential trend of patients with COVID-19 by comparing the neural network prediction models (NN) and ARIMA [1], they were able to predict the incidence of the disease if the previous pattern of disease spread is repeated [36]. A COVID-19 disease prediction study was performed using a machine learning approach. This study proposes a hybrid machine learning method for COVID-19 prediction, using data from Hungary and examining its applicability potential [37]. A study was conducted to predict the spread of COVID-19 using daily data from machine learning and regression methods in India. Social distancing, curfew, and quarantine policies were introduced as critical factors in suppressing the transmission of COVID-19 [38]. The factors associated with death in patients with COVID-19 were investigated in a statistical approach and post-regression analysis. Old age, diabetes, hypertension, kidney disorders, and cardiovascular disease were cited as the main factors in increasing death in COVID-19 patients [39]. In a study on the prediction of COVID-19 in Iran, linear regression was used to estimate the number of positive cases of COVID-19 [40]. In Brazil, they combined the particle filter (PF) method with the SIRU [2] base model to detect and predict the disease from February to September 2020. According to studies, the disease will reach a peak of 25,000 new cases in mid-June 2020 [41]. Univariate analysis and multiple logistic regression were used to investigate the factors predicting COVID-19 [42] in Iran.  Table 2 summarizes the articles reviewed in this section. A paper presents a two-part stochastic modeling procedure that explores the COVID-19 pandemic and the concurrent economic situation as functions of historical pandemic data and mobility control. This approach allows the formulation of an efficient social distancing policy as a stochastic feedback control problem that minimizes the aggregated risks of disease transmission and economic volatility. Furthermore, this study has presented the use of a deep learning algorithm to solve this control problem. Finally, by applying that framework to U.S. data, we empirically examine the efficiency of the U.S. social distancing policy [44]. The effects of coronavirus disease on the Iranian economy are examined with a systems dynamics approach. First, the relationships of important variables affecting GDP in SPSS software are obtained and then the data are analyzed using Vensim software. [3] In this study, we present a system dynamics model to investigate the effects of various factors on the prevalence of COVID-19 and ways to control or reduce transmission and infection. Reviewing the literature on this subject, we found many research gaps that require the attention of researchers. An existing study gap is a lack of studies on the effects of hospital bed capacity limitations and hospital medical staffing on the epidemic system. The proposed model examines the effects of some of the policies announced by the WHO on controlling the transfer rate, the impact of workplace closures, and the allocation of supportive income to reduce economic pressure on population density at the community level. Also, worldwide vaccination and its commencement in Iran, the effect of vaccination, and the influential factors in the vaccine injection rate of the model are investigated. Vaccine availability, people's thinking pressure, and current patient deductions affect vaccination rates. The effectiveness of general vaccination on R0 will also be evaluated. The data for this study came from official sources, including the World Health Organization, the Iranian Ministry of Health and Medical Education, and other relevant literature. With the emergence of a new variant and the coincidence with the decision to reopen schools and universities and reduce restrictions, we examine the situation by considering the booster dose injection. With the previous corona wave in Iran dying out, normalization, and reduced compliance with health protocols, the occurrence of the sixth peak is predicted by examining different scenarios. To prevent the country from entering this stage, encouraging public vaccination and observing health principles, informing the population who resist vaccination, and educating and informing the public in the national media are among the strategies in this study.

## 4. Methodology

System dynamics is a method for modeling and simulating complex systems. In defining this approach, the creator of the systems dynamics method states that the system dynamics method studies data feedback characteristics to prove how the organization interacts structurally, develops policies, delays actions and decisions, and influences success within the organization [45]. From another perspective, system dynamics is used as a way to optimize learning in complex systems. Based on the definitions of systems dynamics, the method is used to study many issues, including industry, economics, and health services [46]. Because the outbreak of the new coronavirus disease has complex and unpredictable behaviors and is strongly influenced by human behavior, modeling the prevalence of COVID-19 using systems dynamics allows us to examine the effect of control parameters on its prevalence. By means of systems dynamics, this paper looks into the factors that affect the spread of the disease and how it is controlled.

In this research, first, by studying the basic model and discovering the existing gaps, the vaccination issue is selected to complete and develop the model. Second, the current behavioral theories such as population aggregation and population density that lead to epidemics and many consequences such as increasing the infection rate are examined. Also, fixed or auxiliary parameters are added to the model as needed to make the model more adaptable to the real world. The structure is plotted based on data from the IRI Ministry of Health and WHO databases based on flow diagrams of crucial variables and reference behaviors. Third, the epidemic simulation model is formulated. Then, the model's validity and its behavioral process are studied. In addition, the model's sensitivity will be analyzed by changing the model parameters, initial conditions, and boundaries. Last, different scenarios are used to look at how to stop diseases, how the model responds to changes in feedback, and what happens as a result. The primary variables in this study include death rate, infection rate, morbidity rate, hospital bed capacity, available staff, and vaccination rate over a 210-day horizon from June 22, 2021. The primary purpose of this study was to investigate the interventions of policymakers, including general education to comply with health protocols, informing the community about the COVID-19 disease to control the prevalence of the disease; the time to see a doctor in case of infection; and extensive vaccination of the population.

## 5. Problem Definition

In response to the outbreak of the coronavirus disease in February 2020, strategic decision-makers in every country, including Iran, endeavored to reduce the transmission of the disease by temporarily closing educational centers and reducing office hours. They also raised community awareness about the disease through the media and introduced ways to prevent and fight against it. At the beginning of the outbreak, these measures could control the prevalence rate of the disease to some extent. However, the country entered a new peak of epidemics within a short time due to the lack of a comprehensive plan for control and prevention policies. Figure 3 shows that the number of infections has been rising at an exponential rate since September 2020. The average number of infections will be highest in mid-August 2021, when there are over 39,000 cases per day.

Based on Figure 6, the number of daily COVID-19 patients in Iran in mid-August 2021 reached more than 38000 people per day. Also, according to Figure 7, the number of COVID-19 deaths in mid-August 2021 reached more than 540 people per day. What can be concluded from this situation is that without principled and coherent planning, government intervention cannot produce accurate future outcomes in controlling the disease. For example, public quarantine reduces people's contact with job closures, but without supportive income, it creates social and economic crises in the long run. The implementation of quarantine policies without considering the relevant protection aspects will lead to its nonacceptance in the long term.

On the other hand, people's risky behaviors and the use of personal protective equipment (PPE) effectively prevent the spread of the disease. Therefore, fighting against this disease is considered a joint project between the people and the political government [28]. With a considerable delay compared to developed countries, vaccination was implemented in Iran in February 2021 as a radical solution alongside interim policies.  Figure 8 compares vaccination trends in Iran, Asia, and the world. As can be seen, the vaccination process in Asia is very similar to the world, but the vaccination pattern in Iran does not match the situation on the continent. There can be different reasons for this deviation. The most important thing is to note that the vaccination process registered in Asia and the world portrays the overall picture of vaccination in all countries. Therefore, the vaccination process in Iran presents a relatively similar pattern that somewhat differs from the vaccination process in a particular country.

Figure 9 compares the daily vaccination rates in Iran and neighboring countries, Turkey and Pakistan. In general, the vaccination situation in Iran is lower than in Pakistan and Turkey. This issue can have several reasons, including delays in the start of the vaccine injection process in Iran due to several reasons, such as sanctions and delays in the clearance of equipment related to mass production of vaccines, barriers to vaccine imports, and so on. It is noteworthy that since many people receive more than one dose of vaccine, this chart does not necessarily correspond to the number of vaccinated individuals.  Figure 10 compares the daily death rate in Iran and neighboring countries, Turkey and Pakistan, since mid-January 2021. As can be seen, on average, the daily death rate in Iran is higher than in neighboring countries.

Comparing the vaccination process and the death rate in Iran and neighboring countries, it is inferred that vaccination as a core solution can significantly reduce death. Nonetheless, it is necessary to prove this position accurately and scientifically by presenting a simulation model. Also, according to the studied information and diagrams, it is necessary to design a model under the conditions of the country to study the behavior of the virus in the presence of vaccination in Iran. Therefore, in this study, the effect of vaccination has been considered to offer an efficient model.

To reduce the number of daily confirmed deaths in Iran, the government decided to reopen most of the public places. After near completion of the fifth wave of COVID-19 in Iran, the reopening of the educational centers was done. Public places such as dormitories, hotels, cinemas, theaters, and gyms reopened and started their activities again. On the other hand, with the introduction of a new variant of the disease called Omicron and the possibility of the formation of the sixth wave of COVID-19, concerns about releasing of restrictions have increased. According to the Health Ministry of Iran, compliance with health protocols is less than 45%; this rate is not the same in all parts of the country; in some parts, compliance with protocols is up to 60%, and in some other cities is less than 40%. The release of the restrictions by the government has made people consider that this disease is over and it is okay to give up the protocols. In such cases, the injection of the third dose as a reminder dose seems necessary and useful to control mortality due to the introduction of the new variant because the government can no longer continue to lockdown and close the offices and the public.

### 5.1. The Basic Model

The effective parameters in the disease outbreak process are determined through reliable scientific sources and medical evidence involved in the crisis. Specific categories of models related to epidemiological articles have formed models. These models are used to describe the prevalence of infectious and epidemic diseases. Their approach was laid out by Ross, Hammer, McKendrick, and Kermack from 1900 to 1935 [47]. In this model, members of a host population are categorized based on their disease status or other characteristics. A change in the value of each characteristic is described as a dynamic system. In this type of model, members of a host population are categorized based on their disease status or other characteristics, and a change in the value of each characteristic is described as a dynamic system [48]. One of these models is the SEIR model, the diagram of which is shown in Figure 11. This model is a modified version of the Kermack and McCendrick (1927) SIR model [49]. It is known as the world's primary epidemic model. In this paper, we considered the SEIR model as the core of the base model. Then, according to the modeling algorithm described, we developed and completed the model until the proposed model was created. The SEIR model comprises four variables:

1. Susceptible individuals: due to the nature of the disease, we consider the initial population, which is assumed to be the total current population of Iran on a scale of one-thousandth, as susceptible individuals, which is deducted from this accumulation rate in the basic model.
2. Exposure individuals: there is an accumulation of the rate of people at risk of infection, but the number of patients decreases with the help of the disease progression rate.
3. Infected individuals: the accumulation of infected individuals entering the country (importing infected) and the rate of disease progression (Advancing) mean eventually becoming infected. However, the rate of recovery and the number of deaths reduce this accumulation.
4. Recovered individuals: it is the accumulation of the number of people whose disease is eliminated by the course of recovery.

At the end of the SEIR model diagram, affected individuals are divided into dead populations (Dying) and recovery populations (Recovering) through the two variables, recovery rate and death rate (Deaths). In the process, active patients (active infected) can infect new people. Relative risk behaviors, initial uncontrolled transmission rate, deduction of susceptible individuals (fraction susceptible), and population density (relative contact density) affect the transmission rate.

The greater the number of patients, the greater the number of patients with severe conditions (serious cases), increasing the pressure on the medical center (hospital strain). Capacity constraints affect the pressure on medical centers, and thus, influence the death rate. The influx of infected people entering the country increases the total number of infected people.

### 5.2. The Developed Model

As mentioned earlier, policies such as quarantine, job closures, and personal protective equipment are acceptable as a short-term solution because, in the long run, these policies are very costly and practically impossible for the government and the people. So, to get rid of the cause of the outbreak, we need a fundamental solution that works for a long time.

This study aimed to investigate the factors affecting the prevalence of the COVID-19 virus and methods to control the spread of the pandemic. Various gaps were observed in the published literature on the factors affecting the spread of the coronavirus disease during the worldwide pandemic. Our proposed model was presented to adapt the model to real-world conditions and investigate the effect of vaccination on the epidemic. The stock-flow diagram of the developed model will be described in the following.

Equitable access to safe and effective vaccines is critical to ending the COVID-19 pandemic, so different countries have begun to immunize themselves through vaccination by studying and researching vaccine production. The WHO emphasizes that vaccination does not mean immunity to disease if exposed to the disease, especially since research is still ongoing on how vaccines protect against disease and infection and transmission. Therefore, masks, hygienic hand disinfection, ensuring proper ventilation inside the house, observing physical distancing, and avoiding crowds are still mandatory. According to the WHO, about 9.37 billion doses of the vaccine were injected worldwide on January 17, 2022. Vaccination-related data in Iran from the date of vaccination (i.e., February 9, 2021) to January 17, 2022, can be reviewed in Table 3 (IRI Ministry of Health and Medical Education).

#### 5.2.1. Vaccination Rate

Three factors directly affect the vaccination rate.

1. Public thinking pressure: the type of opinion people have about the vaccine is very effective in agreeing and disagreeing with the vaccine and, consequently, the vaccination rate. Having a mental background, the type of advertising that people are exposed to, the level of education and awareness, and culture are among the factors that generally shape the type of view people have about receiving the vaccination. As the death toll rises, so does the community's demand for the vaccine. Considering an index between 0 and 1, we applied the effect of this qualitative parameter on the vaccination rate.
2. Vaccine availability: the most critical factor influencing the vaccination rate is its availability, which according to the current situation in which the model is being studied; this amount cannot be more than the demand. So, the least access equals zero, and the maximum will equal the existing demand, which we also considered an index between 0 and 1.
3. Vaccine imports: in the current situation, the import of vaccines is a valid policy due to the need for a rapid increase in vaccination rates and insufficient domestic production. Therefore, the model considered this parameter as an indicator with a value between 0 and 1.

#### 5.2.2. Fraction Infected

Apart from the two factors mentioned above, the number of infected individuals concerning the total number of susceptible individuals affects the vaccination rate, which we considered through a variable called fraction infected, which is equal to the ratio of patients to people exposed to the disease. As the incidence rate increases, the vaccination rate decreases by a ratio.

#### 5.2.3. Vaccinated People

This variable determines the number of people protected by vaccination.

#### 5.2.4. Total Recovered

The number of recovered people is calculated from the number vaccinated and recovered from the disease.

#### 5.2.5. Economic Strain

Another topic of discussion in this article is to examine the effect of economic pressure on the presence of people in the workplace, thus changing the disease transmission rate. The WHO database examines the anticoronavirus disease policies used by different countries in the form of measurable indicators. In this model, we examined the effect of two indicators entitled supportive incomes allocated to the people on the amount of economic pressure due to the pandemic crisis and the impact of job closures on reducing the disease transmission rate.

#### 5.2.6. Working Place Closing

The disease transmission rate decreases with the closure of various offices and occupations.

An article states that vaccination of more than half of the population reduces the person-to-person transmission of the disease to less than half. We applied this reduction as a parameter of the effect of vaccination on reducing R0 (Vaccination effect on reducing R0) and considered the initial value of this reduction as 50% [43].

Income support: paying subsidies to households as supportive income relieves economic pressure on individuals. As a result, people's presence in the workplace, and consequently, the transmission rate is reduced.

Booster Dose: this parameter indicates the percentage of booster dose that increases the overall vaccination rate. Therefore, it is applied as Booster Dose +1 in the vaccination rate formula.

Also, in the developed model, the amount of pressure on medical centers and hospitals and the number of available beds as hospital capacity depends on the number of available nurses (available personnel) and the length of inpatient stay (admission duration). The stock-flow diagram of the proposed model is shown in Figure 12.

The presented model has been compiled using real data obtained from Ministry of Health and Education website and referring to the data and formulas of previous research studies. Also, in the validation section of the text, the validity of the model has been verified by analyzing the sensitivity of key parameters and checking the results. Due to the validity of the data and formulas used and the random selection of the studied time period, as well as the verification of the model by creating different scenarios, the model is valid and applicable to predict the behavior of other pandemics. The references of the formulas are papers [28, 50].

### 5.3. Working Method and Data

Given the high data mining capabilities in data analysis and the use of raw data and the predictive value of data mining, it can be helpful in controlling the quality of statistical data [51]. In solving the proposed model, information about some parameters and influential variables in the problem is considered without any modifications from the basic paper [50]. Also, information about the parameters that externally affect the model is collected from reliable sources and used under the model scale. Given that we are still witnessing the prevalence of COVID-19 at the time of publication of this article, the data used in the new parameters are constantly changing. Therefore, to obtain this information, the data available on the WHO and the IRI Ministry of Health websites and the estimates of the current data trend have been used. According to the latest data available on the WHO website, the population of Iran is about 84 million people, which on a scale of one-thousandth, we considered 84,000. Also, according to the WHO, the number of nurses and beds available in Iran is equal to 21.3 people and 16.2 beds per ten thousand people, which we calculated per 84,000 people. Indicators related to supportive income and job closures are also taken from the WHO website with the values mentioned in the table.

After developing the system dynamics model based on SEIR models and formulating the problem, Vensim software was used to implement the model. The model was calibrated after validation, and its input parameters were analyzed by developing different scenarios. In this step, by examining the values of the target variables to the changes of the input variables, the model's sensitivity to each of the input variables was investigated. Further in this section, information about the new variable formulas added to the model or previous variables whose formula has been updated following the development of existing parameters is presented.

(1) $$\begin{array}{c} R0=3.3-STEP\left(3.3*Vaccination\;effect\;on\;reducing\;R0,40\right)\text{,}\\ Relative\;Contact\;Density=\frac{1}{\left(1+Contact\;Density\;Decline*\left(1-Fraction\;Susceptible\right)\right)}\text{,}\\ Transmission\;Rate=\left(Initial\;Uncontrolled\;Transmission\;Rate*Relative\;Behavioral\;Risk*Fraction\;Susceptible*Relative\;Contact\;Density*\left(1-\frac{Working\;placeclosing}{1000}\right)\right)\text{,}\\ Susceptible=Integ\left(-Infecting-Vaccination\;rate\right),Initial,=InitialPopulation\text{,}\\ Hospital\;Strain=\left(\frac{Serious\;Cases*Admission\;rate}{\left(Hospital\;Capacity*Available\;Personnel\right)}\right)\text{,}\\ Vaccination\;rate=\frac{\left(\left(2+Import\right)*vaccine\;availability*\left(1+people\;thinking\;pressure\right)*\left(1+Booster\;Dose\right)\right)}{\left(1+fractioninfected\right)}\text{,}\\ Vaccinated\;people=Integ\left(Vaccination\;Rate\right),Initial,=40\text{,}\\ Economic\;strain=1-\left(\frac{Income\;Support}{500}\right)\text{,}\\ Total\;recovered=Recovered+Vaccinated\;People\text{,}\\ Vaccination\;effect\;on\;reducing\;R0=0.5\text{,}\\ Vaccine\;Availability=0.9\text{,}\\ Booster\;Dose=STEP\left(0.1,120\right)+STEP\left(0.2,150\right)+STEP\left(0.4,210\right)\text{.} \end{array}$$

## 6. Validation

The validity of the results of studies based on system dynamics depends on the validity of their models [52]. To achieve this goal, a model should present real-world problems more simply so that some real-world variables and structures are eliminated. Hence, it is necessary to check the model's validity to establish that the designed model can provide practical results. There are different methods for validating models of system dynamics. For this purpose, we will refer to two standard methods of comparison with historical data and limit behavior tests in this study. In the first method, we compare the trend of the model results with historical data. If the trends are the same, we can rely on the model results. In the second method, we examine the model under certain conditions. If the model behaves appropriately in these conditions, we can be assured of its accuracy.

Figure13 represented the validity of the proposed model in Vansim software.

### 6.1. Comparison with Historical Data

One method for analyzing the model's validity is to compare the results of implementing the proposed stock-flow diagram with historical data. In this study, if the trend of the graphs is the same, it can be concluded that the model is valid, and it is possible to plan and provide a solution based on the predicted results. Accordingly, in this study, historical data are used to analyze the model behavior in order to demonstrate the validity of the developed model. The results of the model are compared with historical data in the following section. The considered model review period is seven months, from the beginning of summer, from June 29, 2021, to January 25, 2022. The fifth wave of the coronavirus disease pandemic in Iran happened during the time frame given.

Figure 14 shows the vaccinated population resulting from the implementation of the proposed model. As can be seen, there is an upward trend in the growth of the vaccinated population by the end of the year.

Figure 15 shows the vaccinated population in Iran from the start of vaccination by January 5. By comparing Figures 14 and 15, the incremental trend of the graphs promises the model's validity.

The number of patients resulting from implementing the developed model is shown in Figure 16. The peak of this chart is on the 30th day, with the highest number of patients on this day. The behavioral pattern of the diagram follows the overshoot and collapse pattern.

Figure 17 shows the coronavirus disease incidence rate since its outbreak. The fifth peak point in the diagram represents the fifth pandemic wave in Iran. The model's validity is shown by comparing the graphs of vaccinated people and the COVID-19 patients with related historical data and observing the same trend in the graphs in the period from June 29, 2021 to January 25, 2022. Therefore, one can rely on the model's results and act on the proposed policies to control the pandemic. Figure 16 shows the peak points of the coronavirus disease peaks, which have the highest incidence and death rates. Activating the balancing loops in the model prevents the increasing trend of the number of deaths from diverging to infinity. It can be said that the chart trend follows the overshoot and collapse pattern. The bearing capacity decreases over time in the leaps and bounds pattern. As can be seen in the historical data graphs, these graphs follow an oscillating pattern. So, adjustment loops like hospitals, vaccines, people following health rules, etc., keep the graph from going off in a different direction toward infinity.

### 6.2. Extreme Condition Test

The purpose of the limit behavioral test is to examine the model in limit conditions. Based on this test, the values of some parameters are set according to their upper and lower boundaries, and the model is executed. This test shows how the model behaves under certain conditions. If the test results are in line with expectations, we can be assured of the model's reliability. In this test, we have examined the transfer rate variable (R0) under limit conditions. We expect the death rate to increase as the rate of disease transmission increases. By entering different values of this parameter according to Table 4 and implementing the model, the results show that the death rate increases with an increased transmission rate, and with a decreasing transmission rate, the death rate also decreases. The transmission rate for coronavirus disease is 3.3.  Figure 18 shows the death trend concerning different transmission rates.

In the other limit behavior test, the values of public thinking pressure parameters, income support, admission duration, vaccine availability, and workplace closing were changed in the three conditions: worst, normal, and best. The values of the three modes defined are presented in Table 5. In the first case, when all parameters are in the worst condition, we expect the death rate to increase and the number of recovered and vaccinated populations to decrease. In the third case, which is the best case, we expect the death trend, the number of patients, and the number of vaccinated people to be the opposite of what they were in the first case, and we do see a big drop in the death trend.

Figures 19–21 show the model implementation results based on three conditions, namely, pessimistic, normal, and optimistic conditions of death, patients, and vaccinated people. In the first case, with the simultaneous reduction of the values of the parameters, the number of patients increases, and consequently, the vaccination decreases, and the death rate also increases. The third condition, which is better than normal, increases death and morbidity and increases vaccination. Based on the diagram trend in Figures 19–21, the model implementation results align with our expectations.

## 7. Results

### 7.1. Sensitivity Analysis

The purpose of sensitivity analysis is to examine and analyze the variables that have the most significant impact on the model results. In the proposed model, the effect of these changes on death and recovery is examined by changing the value of the behavioral risk variable. These changes in the vaccinated population are also evaluated by considering different values for the parameters affecting vaccination, such as public opinion pressure and vaccine availability.

The behavioral risk variable values for sensitivity analysis are 0, 0.3, 0.5, 0.7, and 1 for the first to fifth case scenarios, respectively. As shown in Figure 19, the more people take care of their health, the lower the death rate. Therefore, based on the death chart in Figure 22, we conclude that the behavioral risk variable significantly affects death and epidemic control. Therefore, the government can devise appropriate policies to encourage people to observe hygienic protocols such as the use of masks and social distancing to prevent further outbreaks of the disease. The curfew policy can also have a good effect as one of the appropriate policies in this area.

Since vaccination is the shortest route to increase immunity against acute COVID-19, we investigate the five different modes of sensitivity of vaccine-dependent variables by changing the numerical value of public thinking pressure parameters and the vaccine availability that affects vaccination rate. The sensitivity of the vaccinated population was evaluated by considering the values of people thinking pressure and vaccine availability as 0, 0.2, 0.5, 0.7, and 1 simultaneously. Given that vaccine availability and public thinking pressure have a positive relationship with the variable of vaccination rate, increasing access to vaccine and public thinking pressure increases. For this reason, in Figure 23, by increasing the values of the two auxiliary variables, the vaccinated population variable has increased. As a result, to increase the vaccinated population, it is necessary to influence its affecting variables. In general, to change a state variable, we need to change its associated rate variables; thus, a state variable cannot be changed directly.

### 7.2. Scenarios

In this article, we have examined different scenarios to examine the possible trends of the coronavirus disease in Iran. Also, we should be ready to face the new conditions in the event of any of the scenarios. In this section, we consider five scenarios.

**Scenario 1 .**

In this scenario, we examine the diffusion of the omicron variant. One of the most critical features of this variant is its high transfer rate, which increases the transfer rate variable. This scenario reflects the actual situation of the community in which the vaccination process, especially the injection of the third dose, the observance of health protocols, and other parameters in the model are based on the actual values in the target community. The purpose of designing this scenario is to show Corona's progress in the real world and compare other plans with this one.

**Scenario 2 .**

The second scenario is based on the observance of hygienic principles and adherence to restrictive laws by the people. As the onset of the sixth wave of the disease intensifies, the government enforces strict laws to force people to observe hygienic principles, wear masks, and prevent ceremonies and gatherings. One of the most critical communities mentioned in the instruction is face-to-face education centers. At the same time, the other parameters of the model remain unchanged.

**Scenario 3 .**

In this scenario, according to statistics published by the Ministry of Health, almost 40% of the population follows health protocols, and due to the increase in patients and increasing public pressure on the government, the speed of vaccination and the process of injecting the third dose will increase. It finds that the government is put under this kind of pressure through cyberspace or other means.

**Scenario 4 .**

This scenario shows that most people in the community follow the health instructions, vaccination is done at the highest rate per day, and the government's financial support is improved. Since adherence to hygiene principles and vaccination is a significant factor in reducing the incidence and mortality rate, we expect the incidence rate to decrease significantly in this scenario. As the number of patients decreases, hospitals will face less pressure, which will allow them to provide better services. This scenario is considered an ideal scenario.

**Scenario 5 .**

The declining trend in compliance with health protocols and the release of some restrictions in the country have unfortunately paved the way for the sixth wave of corona. This scenario is specific to compliance with health protocols and the relaxation of restrictions. In this scenario, educational centers and business districts are opened. The daily contact of people increases, which is due to the release of regulations; on the other hand, injecting the third dose continues to work faster.

Therefore, the import of vaccines in their place is of particular importance and should be given the utmost attention. Of course, the increase in vaccination should not prevent the observance of health protocols, for which, in addition to importing and increasing the speed of vaccines in this scenario, we also increase the variable of contact density decline in society.

### 7.3. Scenario Analysis

In this study, vaccination and adherence to health protocols, considered variables of behavioral risks, have been introduced as two critical factors in reducing the prevalence and incidence. Hygiene is the most important and least expensive way to prevent a COVID-19 infection. The prevalence rate increases as the use of masks, handwashing, and social distancing decreases. The infection and death rates decrease with proper hygiene. The vaccine is also considered one of the essential tools to control COVID-19, which requires more accurate and precise planning for timely injection. According to published statistics from other countries that promptly started general vaccination, the inpatient and death rates have significantly decreased. In Iran, the country faced challenges due to the late completion of domestic vaccine production tests, sanctions, and the lack oftimely import of vaccines. The fourth wave in Iran started at the beginning of April 2021 and then quickly reached its fifth peak with the arrival of the Delta variant at the beginning of the summer of 2021. Due to the unavailability of the required vaccine, the vacancies in the hospitals were quickly replenished, and the death toll increased dramatically. Nonetheless, the government could have prevented the fourth and fifth waves with proper planning, timely imports, and access to vaccines. Despite many problems, vaccination in the country increased from September, and after 5 months, the vaccinated population reached over 60%. Due to concerns about the spread of the new type of Omicron, the booster dose has been included in the WHO program due to the high rate of infection. So, in the last section, different scenarios were set up to look at the status of COVID-19 control and infection under different vaccination and hygiene conditions. The results of these scenarios are shown in Figure 24.

In the first scenario, R0 for the Omicron variant is assumed to be 3.9. In general, the amount of hygiene has decreased from about 80% to about 45% compared to last year, which has increased the incidence of the disease. As we have seen, even in societies where widespread vaccination has taken place, there is still an emphasis on health protocols, mask use, and social distancing. However, despite the Omicron mutation infecting the entire country of Iran, people do not use the mask well, travel, and participate in community gatherings. Therefore, in such circumstances, an increase in infection and death rates is inevitable. Escaping this crisis requires the cooperation of the government and the people. The government should help the vulnerable by creating appropriate conditions for individuals by making timely decisions and adjusting the proper restrictions. By following health rules, people can also play an important role in breaking the chain of infection.

In the second scenario, in contrast to the first, people are forced to follow the health directives of the government, but the vaccination rate is normal. In this scenario, according to Figure 24, it can be seen that the number of patients in this condition has decreased. Scenarios 1 and 2 show the importance of public health principles and the vaccination rate by the government. So, the most important policies that can help control the disease are those that pay attention to behavioral risks, like travel bans, making religious ceremonies and meetings illegal, encouraging health protocols, sending support packages, letting people work from home, and reducing the number of people who take public transportation.

The third scenario is defined based on the conditions of the society in which about 40% of the people in the society follow the health protocols, and the infection and death rate increase sharply. Therefore, public pressure on the government has increased vaccine imports and increased vaccination rates. According to Figure 24, the results of this scenario show that, compared to Scenario 1, the number of patients has gone down as the rate of vaccination has gone up.

In the fourth scenario, in addition to the fact that all members of a society observe health protocols, the vaccination rate is also at its maximum, and supporting people's incomes is also highlighted. Because many people in our society are forced to leave their homes and live in densely populated areas to earn a living, this increases the rate of virus transmission and, consequently, infection and deaths. Hence, one way to stop this trend is for the government to support people's incomes so that they do need to leave home to maintain their livelihood. In this scenario, the transmission rate is reduced by observing the hygienic principles. People are less present in communities due to financial support, and increasing the vaccination rate reduces the incidence of acute illness and death.

Scenario 5 involves discussing the release of some restrictions, such as in-person training. Reducing regulations increases people's contact and therefore increases disease infection between people. With the introduction of the new Omicron variant, the infection rate has increased, doubling the power of disease infection. This scenario clearly shows that nonobservance of health issues causes irreparable damage to public health. Therefore, adhering to the protocols and not releasing restrictions until complete vaccination is achieved should be the government's plan until we reach an acceptable level of safety population to prevent further outbreaks. Also, with the introduction of the omicron variant, the need to increase vaccination and its import is felt more. Therefore, a larger vaccinated population can be reached by importing the vaccine.

### 7.4. Odd Ration

In recent years, odds ratios have been widely used in health studies for the following reasons. First, they provide an estimate (with a confidence interval) for the relationship between two binary variables. Second, they enable us to examine the effects of other variables on that relationship using logistic regression. Thirdly, case studies have a special and very appropriate interpretation. (*∗*A case-control study is a method of designing scientific studies in which the history of independent variables is compared in two groups with a dependent variable (case) and without it (control)) Chance is the ratio of the probability of the event of interest to the probability of its nonoccurrence. It is often estimated as the ratio of the number of times the event of interest occurs to the number of times it does not [53]. Therefore, odds ratio has been used in this study to determine the effect of corona disease on mortality and also to investigate vaccination on mortality.

### 7.5. Investigating the Effect of Corona Disease on Mortality

Odds ratio helps us to obtain the size of the relationship between a specific characteristic with another characteristic in the community and the strength of the relationship between two events [54]. Due to the epidemic crisis of the corona virus disease in different parts of the world and the spread of this disease in Iran from 30th of February 2018 until today, according to the announced statistics, 6,196,721 people out of a population of 84 million people of Iran have been infected with the corona disease during this period, with 132,075 fatalities. To calculate the chance of people dying due to Coronavirus disease and other factors, we need to introduce parameters and values based on the target population, the population of Iran. The whole population of Iran is considered as the sample size. Corona disease patients are represented with CE parameter and those who died due to this disease are shown with DE parameter. According to the website of the Ministry of Health of Iran, 6,064,646 people recovered completely and remained healthy (HE) and 77,803,279 people did not get this disease (CN), of which 879,607 people died due to various reasons other than Coronavirus disease (DN) and 76,923,672 noncoronavirus people are alive and healthy (HN). This information is summarized in Table 6.

And in Table 7, the population that died due to Corona virus and other factors and the living people are represented separately.

To calculate the chance of people dying due to corona and other factors, we first obtain the percentage of death due to corona disease and the percentage of death due to other factors as follows. The percentage of death due to COVID disease is equal to

(2) $$\begin{array}{c} \frac{D_{E}}{C_{E}}=\frac{132.075}{6.196.721}=0.021=\%2.131\text{.} \end{array}$$

The percentage of noncoronavirus death is also equal to

(3) $$\begin{array}{c} \frac{D_{N}}{C_{N}}=\frac{879.607}{77.803.279}=0.011=\%1.130\text{.} \end{array}$$

The relative risk obtained from the difference between these two ratios is equal to

(4) $$\begin{array}{c} 0.021-0.011=0.010 \end{array}$$

The resulting relative risk is calculated as follows:

(5) $$\begin{array}{c} Relative\;Risk=\frac{D_{E}/D_{E}+H_{E}}{D_{N}/D_{N}+H_{N}}=\frac{D_{E}/C_{E}}{D_{N}/C_{N}}=\frac{0.021}{0.011}=1.909\text{.} \end{array}$$

The odds are different. The probability of death if a person contracts this disease is equal to

(6) $$\begin{array}{c} \frac{D_{E}}{H_{E}}=\frac{132.075}{6.064.646}=0.0217\text{.} \end{array}$$

And, the probability of death if a person does not contract this disease is equal to

(7) $$\begin{array}{c} \frac{D_{N}}{H_{N}}=\frac{879.607}{76.923.672}=0.01143\text{.} \end{array}$$

The odds ratio of these two are equal to

(8) $$\begin{array}{c} Odd\;ratio=\frac{D_{E}/H_{E}}{D_{N}/H_{N}}=\frac{132.075/6.064.646}{879.607/76.923.672}=\frac{0.0217}{0.01143}=1.9\text{.} \end{array}$$

As a result, the probability of death of people with corona disease is 1.9 times the probability of death in noncorona disease.

### 7.6. The Importance of Vaccination and its Effect on the Death Rate of People

According to Table 8, 62,037,154 people from the whole population have injected at least one dose of vaccine (VE), and of these, 11,031 people died as a result of this disease (DV). 62026123 people have received at least one dose of vaccine, but they are healthy and have been spared from the corona virus (*H*_*V*_) And, 21962846 people have not received at least one dose of vaccine. (VN) based on Table 9, 62,5088 people have died (*D*_*d*_). Also, 21,900,338 people have not been vaccinated and are healthy.

The death rate of vaccinated people is equal to

(9) $$\begin{array}{c} \frac{D_{V}}{V_{E}}=\frac{11031}{62037154}=0.000177=\%0.017\text{.} \end{array}$$

The death rate of people not vaccinated is equal to

(10) $$\begin{array}{c} \frac{D_{d}}{V_{N}}=\frac{62508}{21962846}=0.00284=\%0.284\text{.} \end{array}$$

The relative risk obtained from the difference between these two ratios is equal to 0.00284 − 0.000177=0.00266

The resulting relative risk is equal to

(11) $$\begin{array}{c} Relative\;Risk=\frac{D_{d}/D_{N}+H_{d}}{D_{V}/D_{V}+H_{V}}=\frac{D_{d}/V_{N}}{D_{V}/V_{E}}=\frac{0.00284}{0.000177}=0.0626\text{.} \end{array}$$

The odds are different. The probability of death if a person has received at least one dose of the vaccine is equal to

(12) $$\begin{array}{c} \frac{D_{V}}{H_{V}}=\frac{11031}{62026123}=0.000177\text{.} \end{array}$$

And the probability of death if a person has not received at least one dose of the vaccine is equal to

(13) $$\begin{array}{c} \frac{D_{d}}{H_{d}}=\frac{62508}{21900338}=0.00285\text{.} \end{array}$$

The odds ratio of these two are equal to

(14) $$\begin{array}{c} Odd\;ratio=\frac{D_{d}/H_{d}}{D_{V}/H_{V}}=\frac{62508/21900338}{11031/62026123}=\frac{0.00285}{0.000177}=16.1\text{.} \end{array}$$

As a result, the death rate of people who did not receive their vaccine is 16.1 times that of people who did The following Table proposed the variables, formulations, and parameters of the model..

## 8. Discussion

The people and the government must work together to prevent the next wave and control the disease. Based on the defined scenarios, the effect of hygiene and vaccination in different conditions was investigated. Observations and analysis show that reducing risky behavior has a significant effect on reducing the number of patients, and increasing the observance of health protocols increases the impact of vaccination. Today, with its focus on vaccinating individuals, the government has a significant role in controlling the disease by vaccinating all members of society as soon as possible by increasing access to vaccines. In addition to vaccination, one of the most important things to consider is enhancing public awareness about the disease.

In some patients, it is observed that they often visit the hospital after a significant part of the lung is involved and the patient's condition has become more acute. In this case, they mainly require admission to the intensive care unit. Meanwhile, the patient could have been admitted to the hospital for short-term hospitalization and may not require intensive care before the acute phase of the disease. Therefore, it can be said that the national media has not performed well in educating people and has been unable to provide the necessary information about observing health and hygiene principles to coronavirus disease patients. Unfortunately, the national media is one step behind the virtual media in raising awareness and does not convey appropriate information to patients and individuals. Therefore, it is necessary for education in the national media to be more coherent, not only to encourage the use of masks but also to inform the public with more accurate details. In addition, the necessity and importance of observing hygienic principles after vaccination should be clarified. It has also been observed in society that some people refuse to be vaccinated for unscientific reasons. Therefore, it is necessary for the national media, with the help of trusted and specialized people in the IRI Ministry of Health, to increase public trust and proper awareness and encourage people to get vaccinated. Also, according to the data and results of sensitivity analysis and different scenarios, it is necessary to focus on behavioral risk control and vaccination to control and reduce coronavirus disease infections. The government should continue to work to maximize vaccine injections and encourage people to adhere to health directives. Because using a vaccine is the shortest way to recovery, the vaccine can be considered a temporary solution. Therefore, encouraging the implementation of health directives can be regarded as a basic solution, and finally, the two proposed solutions should be considered complementary. The effect of the income support variable on this chart is also unavoidable. With the right solutions, the government can provide adequate support for individuals' incomes during the pandemic. Providing a supportive income to people reduces problems of daily living and compensates for reduced incomes, ultimately reducing illness. Another influential variable in this field is the closure of high-risk jobs markets and public places, including schools, mosques, and sports clubs, which directly deal with the rate of disease transmission. As the transmission rate decreases, the incidence also decreases, which ultimately reduces COVID-19 deaths. However, we must have the necessary infrastructure to take this path. For example, with the closure of educational institutions such as schools and universities, we turn to virtualization, which we observe today. Providing a suitable environment for businesses in cyberspace and telecommuting employees in some jobs can also be on the government's plan to prevent an increase in disease transmission by reducing face-to-face communication.

## 9. Conclusion

Identifying the behavior of a phenomenon and providing an appropriate model for it is a prerequisite for designing interventions that can potentially influence the phenomenon's behavior. The COVID-19 epidemic has plunged the world into a health and economic crisis that is perhaps unprecedented since the 1918 Spanish flu epidemic. The virus was first identified in Wuhan, China, in late 2019 and has spread with multiple mutations worldwide, turning COVID-19 disease into a pandemic. The pandemic was followed by the closure of schools and universities, the banning of rallies, and other social distancing policies in countries to disrupt the transmission of the virus. Many types of research have been done in the literature to understand better the behavior of pandemic diseases such as the coronavirus disease and the relevant, effective policies. One of the approaches to studying the behavioral characteristics of COVID-19 is to use the systems dynamics approach. By developing the basic SEIR model and considering interventions and policies such as vaccination, we investigated the factors affecting the spread and control of the coronavirus disease. The developed model was simulated using Vensim software. The desired parameters and variables were formulated according to previous research. We also used the statistics available from the IRI Ministry of Health and the World Health Organization for model data. In this research, vaccination was modeled, and the effect of vaccination on R0 was investigated. Import of vaccine, accessibility to the vaccine, booster dose injections, supportive income, business closure, and economic pressure were considered. Therefore, the occurrence of the sixth wave due to the reduction of observance of health principles and providing management solutions was predicted.

We designed five scenarios based on different conditions and implemented the model. According to the obtained results, the most critical factors in reducing the prevalence of the disease are reducing the behavioral risks of people and increasing the vaccination rate of the booster dose. Observance of hygienic principles leads to the disruption of the transmission chain, and vaccination increases people's immunity against the acute type of infection. In addition, the closure of businesses and educational centers, along with government support for income, effectively controls and reduces the epidemic, which requires cooperation between the people and the government. The factors affecting the rate of vaccination in this study were examined according to the information provided by the IRI Ministry of Health. Despite fluctuations in the vaccination process in Iran, the vaccination rate and vaccine availability have increased. Based on the experience of the last few months, with the government's efforts to easily access the vaccine and inject a booster dose, it can be predicted that the next peak of the coronavirus disease in Iran will be prevented. Given the community's economic conditions and the government's decision to relax the restrictions, it is necessary to plan appropriately to implement this plan. By teaching people how to practice good hygiene after getting vaccinated, eradicating the disease, and giving everyone all their doses, we can control and reduce the disease and stop it from happening again.

In this study, a single type of vaccine was analyzed; future research could evaluate a variety of vaccines from different brands, which would be a more realistic approach. In addition, some vaccination recipients have unfavorable reactions to the vaccine injected, and they are admitted to a hospital that includes people who are elderly or who are asymptomatic patients with COVID-19 disease. These people, by using a parameter, can be separated from the overall number of improvements [55].

## Figures and Tables

**Figure 1:** Graph of the number of daily vaccinations in Iran from February 2021 to mid-January 2022 (Source: ourworldindata.org).

**Figure 2:** Countries where the Omicron type is identified by the end of 2021 (Source: fortune.com).

**Figure 3:** Speed of transmission of omicron variant in countries.

**Figure 4:** Increased infection rate of COVID-19.

**Figure 5:** Declining rate of COVID-19.

**Figure 6:** The number of daily COVID-19 patients in Iran (Source: ourworldindata.org).

**Figure 7:** The number of daily COVID-19 deaths in Iran.

**Figure 8:** Comparison of daily vaccination rates in Iran, Asia, and the world.

**Figure 9:** Comparison of daily vaccination rates in Iran and neighboring countries (Turkey, Pakistan).

**Figure 10:** Comparison of daily death rates in Iran and neighboring countries (Turkey, Pakistan).

**Figure 11:** The basic SEIR model.

**Figure 12:** Stock-flow diagram of the developed model.

**Figure 13:** Validation of proposed model in Vensim software.

**Figure 14:** Results of the vaccinated population.

**Figure 15:** Historical data of vaccination rate (https://ourworldindata.org/covid-vaccinations?country=IRN).

**Figure 16:** Patient incidence rate results.

**Figure 17:** Historical data on the patient incidence rate (Worldometer website) (https://www.worldometers.info/coronavirus/country/iran/#graph-deaths-daily).

**Figure 18:** Extreme condition test with transmission rate variable.

**Figure 19:** The death rate in the limit behavior test.

**Figure 20:** Number of patients in the limit behavior test.

**Figure 21:** Vaccinated population in the extreme condition test.

**Figure 22:** Sensitivity analysis of the behavioral risks variable.

**Figure 23:** Number of people vaccinated in five cases.

**Figure 24:** The results obtained from the fifth scenarios.

**Table 1:** COVID-19 disease world statistics according to the World Health Organization on January-17-2022 report.

Identified 328,844,451	Fatalities 5,557,893		Recovered 267,726,222
Country	Identified	Fatalities	Recovered
USA	66,995,533	873,564	43,090,644
India	37,380,253	486,482	35,237,461
Brazil	23,006,952	621,099	21,710,831
UK	15,217,280	151,987	11,389,181
France	14,172,384	126,967	9,019,484
Russia	10,803,534	312,320	9,858,615
Turkey	10,457,164	84,758	9,665,504
Germany	7,991,432	116,268	7,000,000
Argentina	7,094,865	118,040	6,081,081
Iran	6,221,033	132,075	6,064,646
Pakistan	1,328,487	29,019	1,263,791

**Table 2:** Existing studies on different approaches to modeling COVID-19.

Method	Article	Approach			Country	Vaccination	
		SEIR model	SIR model	Other approach		Yes	No
System dynamics	[24]	✓		PSO	China		✓
	[27]	✓			Iran		✓
	[11]	✓			China		✓
	[13]		✓		Germany	✓	
	[26]				Spain		✓
	[25]						✓
	[23]				Australia		✓
	[28]	✓			Iran		✓
	[43]	✓			Thailand	✓	
	[29]				Indonesia	✓	

Data mining, artificial intelligence, and blockchain	[32, 35]			ML			✓ ✓
	[37]			ML	Hungary		✓
	[36]			NV-ARIMA	Iran		✓
	[34, 38]			Regression- ML data mining	India, Iran		✓ ✓
	[31, 44]			Deep learning blockchain	U.S.	✓	✓

Mathematical modelling	[16]		✓		Brazil		✓
	[10]			SEQIR	India		✓
	[15]			SUQC	China		✓
	[14]	✓					✓
	[12]	✓	✓		Australia		✓
	[20]				Indonesia		✓

Statistical methods	[40]			Linear regression	Iran		✓
	[41]			PF SIRU-	Brazil		✓
	[39]			Regression			✓
	[42]			Univariate analysis and multiple logistic regression	Iran		✓
SD	This research	✓			Iran	✓	

**Table 3:** Vaccination statistics in Iran until January 17, 2022.

Total injected doses	125, 973, 179
Total first injected doses	60, 321, 108
Total second injected doses	53, 130, 215
Total booster injected doses	12, 521, 856

**Table 4:** Different transmission variable values.

Variable name	Modes					
	1	2	3	4	5	6
Disease transmission rate	1	2	2.5	3.3	3.7	4

**Table 5:** Values of other variables.

Variable name	States		
	1	2	3
People thinking pressure	0.1	0.3	0.7
Income support	5	50	95
Inpatient period	13	10	2
Job closures	5	100	150
Vaccine availability	0.1	0.9	1

**Table 6:** Needed information on odds ratios of the effect of Corona.

*C*_*E*_:	6.196.721	*H*_*E*_:	6.064.646	*D*_*N*_:	879.607
*D*_*E*_:	132.075	*C*_*N*_:	77.803.279	*H*_*N*_:	76.923.672

**Table 7:** The healthy population and those who died due to Corona and other factors.

	Death	Healthy
Coronavirus	132,075	6,064,646
Noncoronavirus	879,607	76,923,672

**Table 8:** Required information on odds ratios for vaccination (Source: Ministry of Health & Medical Education).

V_E_:	62037154	H_V_:	62026123	D_d_:	62508
D_V_:	11031	V_N_:	21962846	H_d_:	21900338

**Table 9:** Healthy population and death due to vaccine (Source: Ministry of Health & Medical Education).

	Death	Healthy
Vaccinated	11031	62026123
Not vaccinated	62508	21900338

**Table 10:** Variables, parameters, and formulation of the model.

Variables	Type	Formulas
Susceptible	Level	INTEG (-infecting-vaccination rate, initial population)
Exposed	Level	INTEG (-infecting-vaccination rate, initial population)
Infected	Level	INTEG (Advancing + importing infected-dying-Recovering, 416)
Recovered	Level	INTEG (Recovering,355)
Deaths	Level	INTEG (Dying,24)
Vaccinated people	Level	INTEG (vaccination rate, 40)
Infecting	Rate	Active Infected *∗* Transmission rate
Advancing	Rate	Exposed/Incubation time
Recovering	Rate	Infected/Infection Duration *∗* (1-Fatality rate)
Dying	Rate	Infected *∗* Fatality Rate/Infection duration
Vaccination rate	Rate	((2+Vaccine import) *∗* vaccine availability *∗* (1+people thinking pressure) *∗* (1 + Booster Dose))/(1 + fraction infected)
Admission duration	Exogenous	10
Available personnel	Exogenous	180
People thinking pressure	Exogenous	0.3
Vaccine import	Exogenous	0.6
Booster dose	Endogenos	STEP(0.1, 120)+STEP(0.2, 150)+STEP(0.4, 210)
Vaccine availability	Exogenous	0.9
Income support	Exogenous	50
Economic strain	Endogenos	1-(Income Support/500)
Vaccination effect on reduce R0	Exogenous	0.3
Working place closing total recovered	Exogenous	100
Total recovered	Endogenos	Vaccinated People + recovered
Fraction susceptible	Endogenos	Susceptible/Initial population
Initial population	Endogenos	84000-(0.0001 *∗* (total recovered-deaths))
Active infected	Endogenos	Infected *∗* (1-Isolation effectiveness)
Behavior reaction time	Exogenous	20
Behavioral risk reduction	Exogenous	0.1
Contact density decline	Exogenous	0
Fatality rate	Endogenos	Untreated fatality Rate + (Treated fatality rate-untreated fatality rate)/(1 + Hospital Strain^ hospital capacity sensitivity)
FINAL TIME	Exogenous	210
Fraction infected	Endogenos	Infected/Susceptible
Fraction requiring hospitalization	Exogenous	0.1
Untreated Fatality rate	Exogenous	0.04
Treated Fatality rate	Exogenous	0.01
Transmission rate	Endogenos	(Initial uncontrolled transmission Rate *∗* Relative behavioral Risk *∗* Fraction susceptible *∗* relative contact Density *∗* (1-working place closing/1000))
TIME STEP	Exogenous	0.125
Serious cases	Exogenous	Infected *∗* Fraction requiring hospitalization
Relative contact density	Endogenos	(1 + economic strain)/(1 + Contact density Decline *∗* (1-Fraction susceptible))
Relative behavioral risk	Endogenos	SMOOTH3(1-STEP(Behavioral risk reduction, import Time),Behavior reaction time)
R0	Endogenos	3.3-STEP(3.3 *∗* Vaccination effect on reduce R0, 40)
Public health strain	Endogenos	Infected/Public health capacity
Public HealthCapacity sensitivity	Exogenous	2
Public health capacity	Exogenous	1000
Potential Isolation effectiveness	Exogenous	0
*N* Imported infections	Exogenous	3
Isolation reaction time	Exogenous	2
Isolation effectiveness	Endogenos	SMOOTH3(STEP(Potential Isolation effectiveness, import Time), Isolation reaction Time)/(1 + Public health Strain^ public health capacity sensitivity)
Initial uncontrolled transmission rate	Endogenos	R0/Infection duration
Initial time	Exogenous	0
Infection duration	Exogenous	10
Incubation time	Exogenous	5
Importing infected	Endogenos	N Imported Infections *∗* PULSE(Import time, TIME STEP)/TIME STEP
Import time	Exogenous	10
Hospital strain	Endogenous	(Serious Cases *∗* Admission duration/(Hospital Capacity *∗* Available personnel))
Hospital capacity sensitivity	Exogenous	2
Hospital capacity	Exogenous	137

## Data Availability

The data used in this study cannot be exposed to outsiders.
